The article "Histone Methyltransferase SETD1A Induces Epithelial-Mesenchymal Transition to Promote Invasion and Metastasis Through Epigenetic Reprogramming of Snail in Gastric Cancer" was retracted in 2025. Reason: concerns about the data.

# Histone Methyltransferase SETD1A Induces Epithelial-Mesenchymal Transition to Promote Invasion and Metastasis Through Epigenetic Reprogramming of Snail in Gastric Cancer

**DOI:** 10.3389/fcell.2021.657888

**Published:** 2021-06-07

**Authors:** Jugang Wu, Hongjuan Chai, Haiyan Shan, Chunpeng Pan, Xin Xu, Wenpei Dong, Jiwei Yu, Yan Gu

**Affiliations:** ^1^Department of General Surgery, Shanghai Ninth People’s Hospital, Shanghai Jiao Tong University School of Medicine, Shanghai, China; ^2^Department of Gynecology and Obstetrics, Shanghai Ninth People’s Hospital, Shanghai Jiao Tong University School of Medicine, Shanghai, China; ^3^Department of Obstetrics and Gynecology, Affiliated Suzhou Hospital of Nanjing Medical University, Suzhou, China

**Keywords:** SETD1A, gastric cancer, metastasis, snail, epigenetic reprogram

## Abstract

Aberrant epigenetic modification induces oncogene expression and promotes cancer development. The histone lysine methyltransferase SETD1A, which specifically methylates histone 3 lysine 4 (H3K4), is involved in tumor growth and metastasis, and its ectopic expression has been detected in aggressive malignancies. Our previous study reported that SETD1A promotes gastric cancer (GC) proliferation and tumorigenesis. However, the function and molecular mechanisms of SETD1A in GC metastasis remain to be elucidated. In this study, we found that overexpression of SETD1A promoted GC migration and invasion, whereas knockdown of SETD1A suppressed GC migration and invasion *in vitro*. Moreover, knockdown of SETD1A suppressed GC epithelial-mesenchymal transition (EMT) by increasing the expression of epithelial marker E-cadherin and decreasing the expression of mesenchymal markers, including N-cadherin, Fibronectin, Vimentin, and α-smooth muscle actin (α-SMA). Mechanistically, knockdown of SETD1A reduced the EMT key transcriptional factor snail expression. SETD1A was recruited to the promoter of snail, where SETD1A could methylate H3K4. However, knockdown of SETD1A decreased the methylation of H3K4 on the snail promoter. Furthermore, SETD1A could be a coactivator of snail to induce EMT gene expression. Rescue of snail restored SETD1A knockdown-induced GC migration and invasion inhibition. In addition, knockdown of SETD1A suppressed GC metastasis *in vivo*. In summary, our data revealed that SETD1A mediated the EMT process and induced metastasis through epigenetic reprogramming of snail.

## Introduction

Gastric cancer (GC) is a highly lethal malignant tumor in the digestive system (Cao et al., 2021; Siegel et al., 2021; Sung et al., 2021). Owing to late diagnosis, local recurrences, and distant metastases, GC patients usually face a poor prognosis (Deng et al., 2011; Cristescu et al., 2015). Inhibition of metastasis can ameliorate GC patients’ prognosis (Obermannova and Lordick, 2017). Therefore, more efforts are mandatorily needed to develop novel GC therapeutic strategies for treatment of GC metastasis.

Epithelial-mesenchymal transition (EMT), first discovered in embryonic development, can induce epithelial cells to acquire a mesenchymal phenotype (Bakir et al., 2020). When EMT occurs, the epithelial cells reduce the expression of the epithelial marker (E-cadherin) and increase the expression of mesenchymal markers [N-cadherin, Vimentin, Fibronectin, and α-smooth muscle actin (α-SMA)] (Kalluri and Weinberg, 2009; Ramesh et al., 2020). EMT represents one of the most lethal features of the tumor, metastasis, and, therefore, determines an attractive therapy target in cancer, including GC, prostate, hepatocellular, and colorectal cancers (Huang et al., 2015; Cheaito et al., 2019, 2020; Abed Kahnamouei et al., 2020; Hu et al., 2020; Ramesh et al., 2020; Wang et al., 2020). Identifying novel mediators of EMT might help in defining new therapeutic targets and, hence, novel potential cancer therapies. In the current study, our aim is to explore novel molecular markers of EMT and reveal the potential mechanism resulting in GC metastasis.

Abnormal epigenetic modification contributes to tumorigenesis. Histone methylation, dynamically controlled by lysine methyltransferases (KMT) and demethylase, displays both transcriptional activation and repression activities (Black et al., 2012; Tajima et al., 2015). It is reported that H3K4 aberrant methylation promotes multiple tumor development (Seligson et al., 2009; Ellinger et al., 2010; Chervona and Costa, 2012; Khan et al., 2015). SETD1A, which methylates H3K4, plays key roles in cancer progression, including in colorectal and breast cancers (Shilatifard, 2012; Salz et al., 2014, 2015; Tajima et al., 2015), and sorafenib resistance (Wu et al., 2020a). Our previous study reported that SETD1A promotes GC tumorigenesis by enhancing glycolysis (Wu et al., 2020b). However, whether SETD1A promotes GC metastasis remains unknown. The aim of this study is to determine the role and potential mechanism of SETD1A in GC metastasis.

In this study, our data demonstrate that SETD1A contributes to GC cell migration, invasion, and metastasis. Moreover, we show that SETD1A induces EMT by epigenetic reprogramming of snail.

## Materials and Methods

### Reagents

Fetal bovine serum (FBS; Cat#10099141), penicillin-streptomycin (Cat#15070063), and TRIzol (Cat#15596018) were purchased from Thermo Fisher Scientific (Waltham, MA, United States). HighGene Transfection reagent (Cat#RM09014) was obtained from abclonal (Wuhan, China). A PrimeScript^TM^ RT reagent Kit with gDNA Eraser (Cat#RR047) was purchased from TAKARA Biotechnology (Dalian, China). TransScript II Green One-Step qRT-PCR SuperMix was obtained from TransGen Biotech (Beijing, China). A SimpleChIP^®^ Enzymatic Chromatin IP Kit (Cat#9003) was obtained from Cell Signaling (Danvers, MA, United States). Polybrene (Cat#HY-112735) and crystal violet (Cat#HY-B0324A) were purchased from MedChemExpress (Shanghai, China). A Dual-Luciferase Reporter Assay kit (Cat#1910) was obtained from Promega (Madison, WI, United States).

The primary antibody against SETD1A (Cat#A300-289A) was obtained from Bethyl (Montgomery, TX, United States). The primary antibodies against E-cadherin (Cat#14472), N-cadherin (Cat#13116), Vimentin (Cat#5741), Fibronectin (Cat #26836), α-SMA (Cat#19245), and β-actin (Cat#3700) were purchased from Cell Signaling (Danvers, MA, United States). The primary antibody against snail (Cat#13099-1-AP) was obtained from Proteintech (Wuhan, China). The primary antibody against H3K4me3 (Cat#ab8580) was purchased from Abcam (Cambridge, United Kingdom).

### Cell Lines

AGS, BGC-823, and HEK293T cells were obtained from the Cell Bank of Type Culture Collection of Chinese Academy of Sciences (Shanghai, China). All the cells were cultured in RPMI1640 or DMEM medium supplementing 10% FBS and 1% penicillin-streptomycin at 37°C and 5% CO_2_ condition.

### Establishment of SETD1A Stable Knockdown Cell Clones

SETD1A knockdown cell clones were established as previously (Wu et al., 2020a). In brief, two lentivirus constructs against SETD1A were established by inserting human SETD1A targeting sequences shSETD1A-1, 5′-GGAAAGAGCCATCGGAAATTT-3′; shSETD1A-2, 5′-GACAACAACGAATGAAATATT-3′ into pll3.7 puro vector plasmid. A scrambled vector was used as control. The lentivirus constructs were transfected into HEK293T cells using HighGene transfection reagent following the manufacturer’s instructions. The viruses were collected at 48–72 h after transfection and centrifuged at 2,500 rpm for 30 min to remove contaminating cells. BGC-823 and AGS cells were transfected with the virus in the presence of 10 μg/mL of polybrene. Puromycin (1 μg/mL) was used to select stable SETD1A-knockdown cell clones. The knockdown efficiency was confirmed by Western blot.

### Cell Migration and Invasion

Modified two-chamber transwell migration and invasion assays were performed to determine GC cell migration and invasion. In brief, SETD1A knockdown and control cells suspended in 200 μL of medium without serum were plated on the upper compartment without (migration) or with (invasion) gel of a 24-well transwell chamber, and 700 μL of medium with serum was in the lower compartment. The cells were cultured 48 h, and the chambers were washed by PBS. Cells in the chamber were fixed with methanol, and the non-traversed cells on the upper surface of the filter were removed. The traversed cells on the lower side of the filter were stained with 0.1% crystal violet and counted.

### Western Blot

The Western blot assay was performed as previously (Wu et al., 2020a,b). In brief, cells were lysed by RIPA buffer and centrifuged, the supernatants were collected for Western blot, and 10∼30 μg proteins were separated and transferred onto PVDF membranes. The membranes were probed with the following primary antibodies: SETD1A, E-cadherin, N-cadherin, Vimentin, Fibronectin, α-SMA, and snail at 4°C overnight. Membranes were then probed with appropriated horseradish peroxidase (HRP)-conjugated secondary antibody and visualized by chemiluminescence.

### Real-Time Quantitative PCR (RT-qPCR)

TRIzol and PrimeScriptTM RT reagent Kit with gDNA Eraser were used to isolate total RNA and synthesize cDNA following the manufacturer’s instructions, respectively. TransScript^®^ II Green One-Step qRT-PCR SuperMix was performed to run RT-qPCR by using a Bio-Rad PCR instrument. The primer sequences were listed as below. SETD1A: forward, 5′-TTGCCATGTCAGGTCCAAAAA-3′, reverse, 5′-CGTACTTA CGGCACATATCCTTC-3′; E-cadherin: forward, 5′-CGAGAG CTACACGTTCACGG-3′, Reverse, 5′-GGGTGTCGAGGGAAA AATAGG-3′; N-cadherin: forward, 5′-TTTGATGGAGGTC TCCTAACACC-3′, reverse, 5′-ACGTTTAACACGTTGGAAA TGTG-3′; Vimentin: forward, 5′-AGTCCACTGAGTACCG GAGAC-3′, reverse, 5′-CATTTCACGCATCTGGCGTTC-3′; Fibronectin: forward, 5′-CGGTGGCTGTCAGTCAAAG-3′, reverse, 5′-AAACCTCGGCTTCCTCCATAA-3′; α-SMA: forward, 5′-GGCATTCACGAGACCACCTAC-3′, reverse, 5′-CGACATGACGTTGTTGGCATAC-3′; Snail: forward, 5′-TC GGAAGCCTAACTACAGCGA-3′, reverse, 5′-AGATGAGCAT TGGCAGCGAG-3′; β-actin: forward, 5′-AGCGAGCATCCCC CAAAGTT-3′, reverse, 5′-GGGCACGAAGGCTCATCATT-3′.

### Luciferase Assay

The promoter reporter vector was transfected into cells using HighGene Transfection reagent following the manufacturer’s instructions. Renilla luciferase vector was used as a transfection efficiency control (Wu et al., 2020b). After 48 h, cells were harvested and luciferase activity was measured using the Dual-Luciferase Reporter Assay system.

### Co-immunoprecipitation Assay

Cells were washed by PBS and lysed with IP lysis buffer (20 mM Tris-HCl pH7.4, 100 Mm NaCl, 1 mM EDTA, 1 mM EGTA, 1% Triton X-100, PMSF) (Horos et al., 2019). Cell lysates were centrifuged, and the supernatant was collected for immunoprecipitation (IP). IP was performed by using SETD1A, Snail antibodies, or control immunoglobulin G (IgG). After extensive washing, precipitates were collected. Proteins were eluted and performed by Western blot assay to analyze the interaction.

### Chromatin Immunoprecipitation (ChIP) Assay

The chromatins of control and SETD1A-knockdown BGC-823 cells were immunoprecipitated by H3K4me3, SETD1A, snail antibodies, or non-specific IgG (Santa Cruz). SimpleChIP Enzymatic Chromatin IP Kit (CST, Cat#9003) was used to purify the ChIP DNA following the manufacturer’s instructions. The corresponding snail and N-cadherin promoter were amplified by RT-qPCR. Primers were listed as follows, snail: forward, 5′-TTCACTTCCTCTGGGAAGTCA-3′, reverse, 5′-CAGCACGTGTGGGGCACTGTACC-3′; N-cadherin: forward, 5′-AGCTGATCCTAGTTTGACTCTG-3′, reverse, 5′-TGGCACTGAGGAATGTCTGAG-3′.

### Lung Metastasis

Male nude mice (4∼6 weeks old) were obtained from SLAC Laboratory Animal Co., Ltd. (Shanghai, China) and maintained in specific pathogen-free facilities at a 12:12 h light-dark cycle with *ad libitum* access to food and water. A total of 10^6^ control or SETD1A knockdown BGC-823 cells were injected into nude mice through tail veins. There are six mice in each group. One month later, the mice were sacrificed, and the lung tissues were collected. All animal experiments were according ethical regulations and approved by the Translational Medical Independent Ethics Committee of Shanghai Ninth People’s Hospital (Shanghai, China).

### Statistical Analysis

All the data were presented as mean ± SD. All the experiments were repeated three or more times independently. Statistically significant differences (*p* < 0.05) were examined using Student’s *t*-test.

## Results

### SETD1A Promotes GC Cell Migration and Invasion

Our previous study demonstrated that SETD1A could promote GC cell proliferation and tumorigenesis (Wu et al., 2020b). Here, we determined the biological role of SETD1A in GC invasion and metastasis. Transwell migration and invasion assays were performed to measure the abilities of GC cancer cell migration and invasion. First, SETD1A cDNAs were transfected into GC cells BGC-803 and AGS to increase the expression of SETD1A and then determine the migration and invasion abilities of BGC-803 and AGS cells. As shown in Figures 1A,B, overexpression of SETD1A increased the migration and invasion abilities of BGC-823 and AGS cells. These results indicate that upregulation of SETD1A could enhance GC cell migration and invasion. Furthermore, SETD1A knockdown was performed to determine whether downregulation of SETD1A suppressed GC migration and invasion. To test this aim, SETD1A stable knockdown cell clones were constructed, and their migration and invasion abilities were determined. As shown in Figures 1C,D, two SETD1A stable knockdown cell clones were selected, and their migration and invasion abilities were markedly reduced inBGC-823 (Figure 1C) and AGS (Figure 1D) cells. These results suggest that knockdown of SETD1A inhibits GC cell migration and invasion. In all, our data demonstrates that SETD1A plays a key role in promoting GC cell migration and invasion.

**FIGURE 1:** SETD1A promotes GC cell migration and invasion. **(A,B)** Overexpression of SETD1A increases BGC-823 **(A)** and AGS **(B)** cell migration and invasion. Data from three replicates are shown as the means ± SD. **p < 0.01, ***p < 0.001, ****p < 0.0001 by Student’s *t*-test. **(C,D)** Downregulation of SETD1A decreases BGC-823 **(C)** and AGS **(D)** cell migration and invasion. Data from three replicates are shown as the means ± SD. ***p < 0.001, ****p < 0.0001 by Student’s *t*-test.

### Knockdown of SETD1A Suppresses EMT

EMT participates in tumor invasion and metastasis (Bakir et al., 2020). To determine whether SETD1A mediated EMT in GC cells, we detected the expression of epithelial marker (E-cadherin) and mesenchymal markers (N-cadherin, Vimentin, Fibronectin, and α-SMA) in SETD1A knockdown GC cells. Consistent with our expectations, the protein and mRNA levels of E-cadherin were increased in SETD1A knockdown BGC-823 (Figures 2A,C) and AGS (Figures 2B,D) cells. However, the protein and mRNA levels of N-cadherin, Vimentin, Fibronectin, and α-SMA were decreased in SETD1A knockdown BGC-823 (Figures 2A,C) and AGS (Figures 2B,D) cells. Furthermore, we tested whether SETD1A regulated the expression of key EMT-related transcriptional factors to mediate EMT. The correlations between SETD1A and some key EMT-related transcriptional factors, including snail1, snail2, twist1, and twist2, were analyzed in GC in TCGA database. There was a positive correlation between SETD1A and snail (Supplementary Figure 1A) but not snail2 (Supplementary Figure 1B), twist1 (Supplementary Figure 1C), or twist2 (Supplementary Figure 1D). Western blot and RT-qPCR results also demonstrate that knockdown of SETD1A reduces the expression of snail in BGC-823 (Figures 2E,G) and AGS (Figures 2F,H) cells. These results mean that SETD1A could suppress EMT by reducing the expression of the key EMT transcriptional factor snail.

**FIGURE 2:** Knockdown of SETD1A suppresses GC cell EMT. **(A,B)** Downregulation of SETD1A increases the protein level of E-cadherin and reduces the protein levels of N-cadherin, vimentin, fibronectin, and α-SMA in BGC-823 **(A)** and AGS **(B)** cells. Data from three replicates are shown as the means ± SD. **(C,D)** Downregulation of SETD1A increased the mRNA level of E-cadherin and reduced the mRNA levels of N-cadherin, vimentin, fibronectin and α-SMA in BGC-823 **(C)** and AGS **(D)** cell. Data from three replicates are shown as the means ± SD. ***p < 0.001, ****p < 0.0001 by Student’s *t*-test. **(E,F)** Downregulation of SETD1A increases the protein level of snail in BGC-823 **(E)** and AGS **(F)** cells. Data from three replicates are shown as the means ± SD. **(G,H)** Downregulation of SETD1A increases the mRNA level of snail in BGC-823 **(G)** and AGS **(H)** cells. Data from three replicates are shown as the means ± SD. ***p < 0.001, ****p < 0.0001 by Student’s *t-*test.

### SETD1A Promotes Snail Expression by Increasing the H3K4me3 Levels on the Snail Promoter

Our results demonstrate that SETD1A mediates the protein and mRNA levels of snail; we hypothesized that SETD1A transcriptionally controlled the expression of snail. To test this hypothesis, the promoter reporter of snail with different amounts of SETD1A expression plasmid were cotransfected into 293T cells, and then the activity of the snail promoter reporter was measured by the luciferase activity assay. SETD1A increased snail promoter reporter activity in a dose-dependent manner (Figure 3A). In addition, downregulation of SETD1A decreased the promoter activity of snail in BGC-823 (Figures 3B,C) AGS cells. Furthermore, we tested whether SETD1A could recruit snail promoter and increase the H3K4me3 levels. The chromatin immunoprecipitation (ChIP) results exhibit that knockdown of SETD1A decreases the recruitments of SETD1A to the promoter of snail (Figure 3D) and reduces H3K4me3 levels on the promoter of snail (Figure 3E) in BGC-823 cells. These results indicate that SETD1A increases the expression of snail at the transcriptional level.

**FIGURE 3:** SETD1A promote snail expression by increasing the H3K4me3 levels on the snail promoter. **(A)** SETD1A enhances the promoter reporter activity of snail in a dose-dependent manner in HEK293T cells. Data from three replicates are shown as the means ± SD. **p < 0.01, ***p < 0.001, ****p < 0.0001 by Student’s *t-*test. **(B,C)** Downregulation of SETD1A decreases the promoter reporter activity of snail in BGC-823 and AGS cells. Data from three replicates are shown as the means ± SD. ***p < 0.001, ****p < 0.0001 by Student’s *t*-test. **(D,E)** Downregulation of SETD1A reduces the levels of SETD1A **(D)** and H3K4me3 **(E)** on the promoter of snail in BGC-823 cells. Data from three replicates are shown as the means ± SD. ****p < 0.0001 by Student’s *t*-test.

### SETD1A Induces EMT Through Coactivation of Snail

We reported that SETD1A could be a coactivator to induce gene expression (Wu et al., 2020b). We propose a hypothesis that SETD1A could be a coactivator of snail to induce EMT gene expression. To test this hypothesis, HEK293T cells were cotransfected with SETD1A and/or snail expression plasmids, together with the N-cadherin promoter reporter, and then the luciferase activity assay was performed. overexpression of SETD1A or snail alone increased the reporter activity threefold or sevenfold, respectively, and the reporter activity reached 25-fold when there was simultaneous overexpression of SETD1A and snail together (Figure 4A). In contrast, knockdown of SETD1A reduced the report activity of N-cadherin in BGC-823 (Figure 4B) and AGS (Figure 4C) cells. Furthermore, we determined whether SETD1A could bind with snail. The co-immunoprecipitation (co-IP) assay using SETD1A and snail antibodies, respectively, was performed to detect the interaction. The interaction between snail and SETD1A could be detected in BGC-823 (Figure 4D) and AGS (Figure 4E) cells. These results suggest that SETD1A could cooperate with snail to induce EMT gene expression. In addition, we also tested whether SETD1A could assist snail to recruit the promoters of snail target EMT genes. The ChIP assay was performed to detect the recruitments. The results show that knockdown of SETD1A reduces the recruitments of SETD1A to the promoter of N-cadherin as expected (Figure 4F); meanwhile, knockdown of SETD1A also markedly decreased H3K4me3 levels (Figure 4G) and snail recruitment (Figure 4H) on the promoter of N-cadherin. These data suggest that SETD1A could increase H3K4me3 levels on the promoter of N-cadherin to facilitate snail transactivation.

**FIGURE 4:** SETD1A induces EMT through coactivation of snail. **(A)** SETD1A cooperates with snail to enhance the promoter reporter activity of N-cadherin. Data from three replicates are shown as the means ± SD. ****p < 0.0001 by Student’s *t*-test. **(B,C)** Downregulation of SETD1A decreases the promoter reporter activity of N-cadherin in BGC-823 and AGS cells. Data from three replicates are shown as the means ± SD. ***p < 0.001, ****p < 0.0001 by Student’s *t*-test. **(D,E)** Co-IP analysis of the interaction between SETD1A and snail. Data from three replicates are shown as the means ± SD. **(F–H)** Downregulation of SETD1A reduced the levels of SETD1A **(F)**, H3K4me3 **(G)**, and snail **(H)** on the promoter of N-cadherin in BGC-823 cells. Data from three replicates are shown as the means ± SD. **p < 0.01, ****p < 0.0001 by Student’s *t*-test.

### Restoration of Snail-Associated EMT Recovers GC Cell Migration and Invasion Inhibited by SETD1A Knockdown

To validate the essential role of snail-associated EMT in SETD1A-induced GC cell migration and invasion, a snail expression plasmid was used to rescue the snail expression in SETD1A knockdown BGC-823 and AGS cells, and then transwell migration and invasion assays were performed to determine the GC cell migration and invasion. The results exhibited that restoration of snail resulted in recovering EMT, cell migration, and invasion suppressed by SETD1A knockdown in BGC-823 (Figure 5A) and AGS (Figure 5B) cells. These results indicate that SETD1A induces EMT and GC cell migration and invasion by enhancing snail associated EMT.

**FIGURE 5:** Restoration of snail-associated EMT recovers GC cell migration and invasion inhibited by SETD1A knockdown. **(A,B)** Restoration of snail resulted in recovering EMT, cell migration, and invasion suppressed by SETD1A knockdown in BGC-823 **(A)** and AGS **(B)** cells. Data from three replicates are shown as the means ± SD. **p < 0.01, ***p < 0.001 by Student’s *t-*test.

### Knockdown of SETD1A in BGC-823 Cells Inhibits Metastasis *in vivo*

Owing to SETD1A playing an essential role in promoting GC cell migration and invasion *in vitro*, we further tested whether SETD1A could also promote GC cell metastasis *in vivo*. SETD1A-knockdown and control BGC-823 cells were injected into nude mice through the tail vein, and the number of tumors in the lung were counted. The number of tumors were fewer in the SETD1A knockdown BGC-823 cells (Figure 6A), and the areas of metastasis were reduced in the SETD1A knockdown BGC-823 cells (Figure 6B). These results suggest that SETD1A promotes GC metastasis *in vivo*.

**FIGURE 6:** Knockdown of SETD1A reduces GC cell metastasis. **(A)** Downregulation of SETD1A in BGC-823 cells reduces the number of tumors in the lung surface. Data from six mice are shown as the means ± SD. ***p < 0.001. **(B)** Downregulation of SETD1A in BGC-823 cells reduces tumor growth in the lung. Data from six mice are shown as the means ± SD. ****p < 0.0001 by Student’s *t*-test.

## Discussion

EMT participates in gastric cancer metastasis. Snail is a key EMT-associated transcription factor, which enhances EMT (Semenza, 2010). Exploiting the mediator that controls snail-associated EMT is important for discovering effective and targeted treatments for cancer metastasis. In the present study, we have confirmed that SETD1A induces EMT to facilitate GC cancer cell migration, invasion, and metastasis by epigenetic reprogramming of snail (Figures 1, 6). Knockdown of SETD1A suppresses EMT and GC cell migration, invasion, and metastasis, accompanied with increased expression of an epithelial marker (E-cadherin) and reduced mesenchymal markers (N-cadherin, Vimentin, Fibronectin, and α-SMA) (Figure 2). Furthermore, restoration of snail-associated EMT by rescuing the expression of snail-recovered GC cell migration and invasion is suppressed by SETD1A knockdown (Figure 5). In all, all these data demonstrate that SETD1A could be a metastasis-related biomarker by inducing snail-associated EMT.

EMT is a biologic process that switches the polarized epithelial phenotype of the cell to a mesenchymal cell phenotype, leading to an increase in migration and invasion capacity and enhancing resistance to apoptosis (Kalluri and Weinberg, 2009; Das et al., 2019). Cancer, being a highly heterogeneous disease known for its accumulations of various abnormalities in the cell, often recapitulates and manipulates the developmental EMT program in a partial and transient fashion to acquire advantageous features for its survival and propagation (Hanahan and Weinberg, 2011). The EMT process is controlled by multiple transcription factors, including Snail, Slug, Twist, an Zeb1/2, which aid enhancing invasive ability, dissemination to distant sites, and metastatic colonization (Brabletz et al., 2018; Williams et al., 2019). To identify the novel mediators of EMT contributes to treating cancer. Increased evidence shows that EMT could be regulated by epigenetic modification, including H3K27/H3K9 methylation, which induces the expression of EMT-related gene expression (Cui et al., 2018; Lai et al., 2020). To identify the novel epigenetic modification mediator of EMT will contribute to discovering the biomarkers and revealing the mechanism of tumor metastasis. In the current study, we discovered that an H3K4 methyltransferase SETD1A could increase the expression of snail by recruiting to and methylating the H3K4 on the promoter of snail and be a coactivator of snail to enhance snail’s transactivation, which induces EMT.

The SET1/MLL H3K4 methyltransferase SETD1A can add mono- to tri-methyl on H3K4 to induce gene expression (Schneider et al., 2005). It is reported that SETD1A is upregulated and promotes cancer development, including breast cancer, lung adenocarcinoma, colorectal cancer, and GC (Salz et al., 2014, 2015; Fang et al., 2018; Jin et al., 2018; Wu et al., 2020b). In the present study, our *in vitro* data demonstrate that SETD1A promotes GC cell migration and invasion (Figure 1). However, we have only used the lung metastasis model to validate that knockdown of SETD1A suppresses GC cell metastasis (Figure 6). Further *in vivo* models will be necessary to fully confirm the function of SETD1A in GC cell metastasis. We reported that patients who expressed high levels of SETD1A faced a poor prognosis in our previous paper (Wu et al., 2020b).

Taken together, the current study indicates that SETD1A plays an essential role in promoting GC invasion and metastasis. This promotion ability may be dependent on the induction of EMT through epigenetic reprogramming of snail (Figure 7).

**FIGURE 7:** Working model: STED1A promotes GC cell migration, invasion, and metastasis through enhancing snail-associated EMT.

## Data Availability Statement

The original contributions presented in the study are included in the article/Supplementary Material, further inquiries can be directed to the corresponding author/s.

## Ethics Statement

The animal study was reviewed and approved by the Translational Medical Independent Ethics Committee of Shanghai Ninth People’s Hospital.

## Author Contributions

YG, JY, and JW contributed to the study concepts, study design, and manuscript edit and review. JW, HC, and HS carried out the study design, most experiments, data acquisition and analysis, and manuscript preparation. CP, XX, and WD performed some cellular experiments, Western blot, and animal experiments. All authors read and approved the final manuscript.

## Conflict of Interest

The authors declare that the research was conducted in the absence of any commercial or financial relationships that could be construed as a potential conflict of interest.

## Supplementary Material

Supplementary Figure 1 The correlation between SETD1A and snail1, snail2, twist1, and twist2 in gastric cancer samples in TCGA database.

Supplementary Figure 2 Uncropped scans of Western blots.
